The article "Long non-coding RNA AK096174 promotes cell proliferation and invasion in gastric cancer by regulating WDR66 expression" was retracted in 2023. Reasons: errors in the materials; errors in the data.

# Long non-coding RNA AK096174 promotes cell proliferation and invasion in gastric cancer by regulating WDR66 expression

**DOI:** 10.1042/BSR20180277

**Published:** 2018-07-18

**Authors:** Yeqian Zhang, Site Yu, Zizhen Zhang, Gang Zhao, Jia Xu

**Affiliations:** Department of Gastrointestinal Surgery, Renji Hospital, School of Medicine, Shanghai Jiao Tong University, Shanghai 200127, P.R. China

**Keywords:** AK096174, Gastric cancer, Invasion, Long noncoding RNA, WD repeat-containing protein

## Abstract

Gastric cancer (GC) is one of the major causes of cancer deaths worldwide; however, the mechanism of carcinogenesis is complex and poorly understood. Long non-coding RNA (lncRNA) has been reported to be involved in the development of multiple cancers. Here, we identified a novel lncRNA, AK096174, which was up-regulated and associated with tumorigenesis, tumor size, metastasis, and poor prognosis in GC. Our data showed that AK096174 was highly expressed in the GC tissues and cell lines (SGC-7901, AGS, BGC-823, MGC-803), and patients with higher AK096174 expression had a poorer prognosis and shorter overall survival (OS). AK096174 knockdown inhibited the proliferation, migration, and invasiveness in SGC-7901 and BGC-823 cells, whereas AK096174 overexpression had the promoting effects. Furthermore, mechanistic investigation showed that AK096174 positively correlated with the expression of WD repeat-containing protein 66 (*WDR66*) gene at the translational level. Knockdown of WRD66 attenuated the positive impact of AK096174 in GC cells. The findings of the present study establish a function for AK096174 in GC progression and suggest it may serve as a potential target for GC therapy in the future.

## Introduction

Gastric cancer (GC) is one of the major causes of cancer deaths worldwide and incidence rates are highest in Eastern Asia including Korea, Japan, and China [1]. Although numerous efforts have been made to improve the diagnosis and survival of GC patients, this disease remains a major challenge due to the limited therapeutic options, tumor metastasis, and recurrence [2,3]. The mechanism of gastric carcinogenesis is complex, and there is still no curative modality for late-diagnosed GC [4,5]. Therefore, it is essential to develop novel diagnostic markers and effective therapeutic targets for GC patients.

Long non-coding RNAs (lncRNAs) are newly identified members of the non-coding RNA family, which are greater than 200 nts in length and lack protein-coding ability [6]. Studies have revealed that lncRNAs regulate gene expression at different levels, including chromatin reprogramming, transcriptional processing, miRNA sponging, and other processes [7]. Growing evidence shows that aberrant expression of lncRNAs can play an important role during the initiation and development of GC [8,9]. For instance, the ectopic lncRNA expression, including that of H19 [10], HOTAIR [11], HOXA11-AS [12], and MALAT1 [13] significantly regulate GC cell proliferation, cell cycle, apoptosis, invasion, migration, metastasis, and tumorigenicity. Although lncRNAs have been found to be involved in various cellular processes, more specific mechanisms of lncRNAs in GC initiation and development need to be further teased out. Furthermore, it remains unclear whether other lncRNAs are also involved in GC tumorigenesis and progression.

The article "Long non-coding RNA AK096174 promotes cell proliferation and invasion in gastric cancer by regulating WDR66 expression" was retracted in 2023. Reasons: errors in the materials; errors in the data.

In the present study, we identified a novel oncogenic lncRNA, AK096174, by microarray analysis and subsequently validated this finding in GC tissue specimens. We found expression of AK096174 to be significantly increased in GC tissues, and patients with high AK096174 expression had poor survival outcomes. Moreover, AK096174 could serve as an independent predictor for overall survival (OS) and disease-free survival (DFS) in GC. Further *in vitro* experiments demonstrated the oncogenic role of AK096174: it promoted cell proliferation, migration, and invasion by interacting with WD repeat-containing protein 66 (WDR66) and enhances its expression at the translational level. Thus, the findings of the present study establish the function of AK096174 in GC progression and suggest its potential as a new target in GC therapy.

## Materials and methods

### Patients and tissue samples

The human GC tissue and paired-adjacent gastric tissue samples used in the present study were obtained from 32 GC patients who underwent surgical resection at Renji Hospital between 2010 and 2016. Clinical and pathological characteristics were obtained from patient charts. All samples were frozen in liquid nitrogen immediately after resection and stored at 80°C until use. Tumor histological grades were assessed according to the criteria set by the World Health Organization (WHO) using the 7th edition TNM staging of the International Union Against Cancer (UICC). The present study was approved by the Ethics Committee of Renji Hospital, and written informed consent was obtained from each patient.

### Microarray analysis

Total RNA from tumor and non-cancerous normal tissues obtained from five GC patients was isolated using the TRIzol reagent (Invitrogen, Carlsbad, CA, U.S.A.), amplified and transcribed into cDNA. The biotinylated cDNA was hybridized to the Human Gene 2.0 ST Array (Affymetrix, Santa Clara, CA, U.S.A.), as performed by Shanghai Kangcheng Biotechnology Co., following the manufacturer’s instructions. The microarray data were analyzed using Transcriptome Analysis Console (TAC) software version 3.0 (Affymetrix).

The article "Long non-coding RNA AK096174 promotes cell proliferation and invasion in gastric cancer by regulating WDR66 expression" was retracted in 2023. Reasons: errors in the materials; errors in the data.

### Cell lines and cell culture

A normal human gastric epithelium cell line (GES-1) and GC cell lines (SGC-7901, MGC-803, MKN-28, AGS, and BGC-823) were purchased from the Institute of Biochemistry and Cell Biology, Chinese Academy of Sciences, Shanghai, China. MGC-803, SGC-7901, MKN-28, and BGC-823 were cultured in RPMI 1640 medium (Invitrogen, Carlsbad, CA, U.S.A.), AGS was cultured in F-12 medium (Invitrogen), and GES-1 was cultured in Dulbecco’s modifed Eagle medium (Invitrogen). All cell culture media were supplemented with 10% FBS, 1% penicillin and streptomycin. The GC cells were maintained in a humidified atmosphere of 5% CO_2_ and 95% air at 37°C. Cell lines were authenticated using Short Tandem Repeat (STR) analysis as described in 2012 in ANSI Standard (ASN-0002) by the ATCC Standards Development Organization (SDO) and in Capes-Davis et al. (Supplementary material).

### Cell transfection

SGC-7901 and BGC-823 cells (2 × 10^5^) were plated in six-well culture plates and incubated for 24 h, then transfected with two si-WDR66 or negative control siRNA (GenePharma, Shanghai, China) using Lipofectamine 2000 (Invitrogen) following the manufacturer’s protocol. Target sequences for WDR66 siRNAs: si-WDR66 1#, Sense: 5′-GUAACUAAGGGUGAGCAUA-3′, si-WDR66 2#, Sense: 5′- GUUACUAAAGGUGAGCAUA-3′. The human AK096174 and WDR66 cDNA sequences were synthesized and then ligated into the pCDNA3.1 vector (Invitrogen, Shanghai, China). AK096174 shRNA oligos were synthesized, annealed, and ligated into the shRNA vector. Plasmid vectors (pCDNA-WDR66, pCDNA-AK096174, sh-AK096174, and empty vector) for transfection were prepared using Midiprep kits (Qiagen, Hilden, Germany). At 48 h post transfection, cells were harvested for qPCR or Western blot analysis. Target sequences for AK096174 shRNAs: sh-AK096174 1#, Sense: 5′-CACCGCCACTCCACCTCAAACTCTTACCTTCGAAAAGGTAAGAGTTTGAGGTGGAGTGG-3′, sh-AK096174 2#, Sense: 5′-CACCGGGTCATTAAGGGTTCAAGCGAACTTGAACAGAGACTCTGTCCCTTAATGACCC-3′.

### Cell proliferation

The capacity for cellular proliferation was measured with the cell counting kit 8 (CCK-8, Beyotime, China). Twenty-four hours after siRNA or vectors transfection, GC cells (approximately 2.5 × 10^3^) were seeded into 96-well culture plates for 24, 48, and 72 h. The cells were then incubated with 10 ml CCK-8 for 1 h at 37°C. The optical density was determined with a spectrophotometer (Spectra Max plus384, Molecular Devices) at a wavelength of 450 nm.

### Cell migration and invasion assays

Twenty-four-well Transwell chambers with 8-μm pore size polycarbonate (Corning Incorporated, Corning, NY, U.S.A) were used for cell migration and invasion assays. For invasion assays, the top side of the membrane was coated with Matrigel (BD Biosciences, Franklin Lakes, NJ, U.S.A), and then 1 × 10^5^ cells (in each well) in serum-free RPMI 1640 medium were seeded on the chambers. RPMI 1640 containing 10% FBS was added to the wells under the chamber. For migration analysis, 5 × 10^4^ cells (in each well) in serum-free RPMI 1640 medium were seeded on to the chambers without Matrigel. After 24 h of incubation, cotton swabs were used to remove the cells inside the upper chamber, while the cells on the other side of the membrane surface were fixed and stained with 0.5% Crystal Violet solution. Five random fields were counted in each well.

The article "Long non-coding RNA AK096174 promotes cell proliferation and invasion in gastric cancer by regulating WDR66 expression" was retracted in 2023. Reasons: errors in the materials; errors in the data.

### RNA extraction and quantitative real-time PCR

Total RNA was extracted from GC tissues and cell lines using TRIzol reagent (Invitrogen). One microgram RNA was reverse transcribed in a final volume of 20  μl using random primers under standard conditions for the PrimeScript RT reagent Kit (TaKaRa, Dalian, China). SYBR Premix ExTaq (TaKaRa) was used to determine AK096174 and WDR66 expression levels, following the manufacturer’s instructions. The expression data of AK096174 and WDR66 were normalized to the expression of U6 or β-actin. The following primers were used: 5′-TCCCACACGACCACAGATACGG-3′ (sense) and 5′-CACCATGCCCTGAGGAGAAC-3′ (antisense) for AK096174; 5′-CAACCTGCTCCGTCAAA-3′ (sense) and 5′-TAAACATTCCTGGTAACTTCAC-3′ (antisense) for WDR66; and 5′-CTCGCTTCGGCAGCACA-3′ (sense) and 5′-AACGCTTCAGGAATTTGCGT-3′ (antisense) for U6; 5′-AGCGAGCATCCCCCAAAGTT-3′ (sense) and 5′-GGGCACGAAGGCTCATCATT-3′ (antisense) for β-actin.

### Western blot

RIPA extraction reagent (Beyotime, Beijing, China) supplemented with protease inhibitor cocktail (Roche, CA, U.S.A.) was used to lyse the BGC-823 and SGC-7901 cells and extract the protein. Then, 40 μg of protein was separated by SDS/PAGE (8–12% gel) and transferred to 0.22-μm PVDF membranes (Millipore). The membrane was blocked for 1 h at room temperature in Tris-phosphate buffer containing 0.1% Tween 20 with 5% skim milk (Sigma-Aldrich, St. Louis, U.S.A.), and subsequently incubated at room temperature for 1–2 h with primary antibodies. Primary antibodies were epithelial marker E-cadherin (1:1000, Abcam); mesenchymal marker N-cadherin (1:1000, Abcam), Snail (1:1000, Cell Signaling Technology), ZEB1 (1:1000, Cell Signaling Technology), and β-actin (1:2000, Abcam). ECL chromogenic substrate was quantitated by densitometry (Quantity One software; Bio-Rad, Hercules, CA, U.S.A.).

### Statistical analysis

All analyzing data for continuous and categorical variables are presented as the mean ± S.E.M. and the number of lesions with the percentage. Student’s *t* test, χ^2^ test, or Wilcoxon’s test was used to analyze the significance of the differences between groups. The Kaplan–Meier method and log-rank test were used for DFS analysis. Statistical analysis was performed using SPSS 17.0 computer software (SPSS Inc., Chicago, IL, U.S.A.), and GraphPad Prism version 5 for Windows (GraphPad Software*). P*<0.05 was considered statistically significant.

The article "Long non-coding RNA AK096174 promotes cell proliferation and invasion in gastric cancer by regulating WDR66 expression" was retracted in 2023. Reasons: errors in the materials; errors in the data.

## Results

### Altered expression of AK096174 in GC cell lines and GC tissues

To screen lncRNAs involved in GC progression, tumor and non-cancerous normal tissues obtained from five GC patients were selected for microarray analysis (Affymetrix GeneChip® Human Gene 2.0). We found 30 lncRNAs showing >two-fold change in tumor tissues compared with normal tissues (15 up-regulated and 15 down-regulated) (Figure 1A). Then, we selected the lncRNA AK096174 with a fold change >4 and validated its expression using quantitative real-time PCR in 32 paired GC and non-cancerous normal tissues. U6 was used as an internal control. The results showed that AK096174 was increased in 62.5% (20/32) of GC tissues compared with normal tissues (Figure 1B,C). Furthermore, compared with normal gastric cell line GES-1, AK096174 exhibited higher expression levels in SGC-7901, BGC-823, MGC-803, and AGS cell lines (Figure 1D). Collectively, these results indicate that AK096174 is up-regulated in GC.

**Figure 1:** Expression of AK096174 was up-regulated in gastric cell lines and tissues (**A**) Cluster maps of top up-regulated or down-regulated lncRNAs in GC tissues compared with matched adjacent tissues (MATs). (**B**,**C**) The relative expression of AK096174 was measured by quantitative real-time PCR in 32 GC tissues and paired adjacent gastric tissues. The expression of AK096174 was calculated with the 2^−ΔΔ*C*^_T_ method using U6 levels for normalization. (**D**) Expression of AK096174 in human normal gastric epithelial cell line GES-1 and five GC cell lines. (**E**) Kaplan–Meier plots show DFS according to the level of AK096174 in patients who underwent surgery. Data are presented as mean ± S.D. Experiments were independently conducted three times to obtain the presented data. *P<0.05 and **P<0.01.

### The expression of AK096174 and clinicopathologic characteristics of GC

Clinicopathologic features were analyzed according to the level of AK096174 expression. The statistical analysis showed that a higher AK096174 level was associated with larger tumors (*P*=0.001), advanced pathological stage *(P*=0.035), and lymph node metastasis (*P*=0.004). However, AK096174 expression level was not related to other factors including gender (*P*=0.706) and age (*P*=0.581) in GC (Table 1). DFS in the low level of AK096174 group tended to be superior to that in the high level of AK096174 group; however, there was no significant statistical difference (*P*=0.184) (Figure 1E).

The article "Long non-coding RNA AK096174 promotes cell proliferation and invasion in gastric cancer by regulating WDR66 expression" was retracted in 2023. Reasons: errors in the materials; errors in the data.

**Table 1:** Expression of AK096174 in 32 GC tissues compared with adjacent normal tissues

Characteristics	Number	AK096174 level				χ^2^	*P*-value
		Lower (*n*=12)		Higher (*n*=20)			
Gender							
Male	20	8 (40.0%)		12 (60.0%)		0.142	0.706
Female	12	4(33.3%)		8 (66.7%)			
Age (years)							
≤60	14	6 (42.9%)		8 (57.1%)		0.305	0.581
>60	18	6 (33.3%)		12 (66.7%)			
Tumor size (cm)							
<5	15	10 (66.7%)		5 (33.3%)		10.248	0.001*
≥5	17	2 (11.8%)		15 (88.2%)			
Differentiation							
Well	5	4 (80.0%)		1 (20.0%)		9.808	0.007*
Moderate	8	5 (62.5%)		3 (37.5%)			
Poor	19	3 (15.8%)		16 (84.2%)			
Lymphovascular invasion							
No	25	10 (40.0%)		15 (60.0%)		0.305	0.581
Yes	7	2 (28.6%)		5 (71.4%)			
Depth of tumor invasion							
T1	3	2	66.7%	1	33.3%	4.306	0.23
T2	6	3	50.0%	3	50.0%		
T3	10	5	50.0%	5	50.0%		
T4	12	2	16.7%	10	83.3%		
Lymph metastasis							
N0	10	8	80.0%	2	20.0%	13.44	0.004*
N1	4	2	50.0%	2	50.0%		
N2	6	1	16.7%	5	83.3%		
N3	12	1	8.3%	11	91.7%		
TNM stage							
I	3	2	66.7%	1	33.3%	6.684	0.035*
II	9	5	55.6%	4	44.4%		
III	20	3	15.0%	17	85.0%		

* Overall <0.05.

### Effect of AK096174 on proliferation, migration, and invasion of GC cells

To investigate the biological function of AK096174 in GC cells, we first performed qPCR analysis to detect the expression of AK096174 in GC cells transfected with sh-AK096174, pCDNA-AK096174, and empty vector. Results of qPCR analysis showed that AK096174 expression was knocked down by ~79% in sh-AK096174 1#-transfected cells and ~74% in sh-AK096174 2#-transfected cells. AK096184 expression was up-regulated by ~37-folds in SGC-7901 cells and ~24-folds in BGC-823 cells in AK096174 overexpression vector-transfected cells when compared with control cells (Figure 2A).

**Figure 2:** The effect of AK096174 on cell proliferation, migration, and invasion in gastric cell lines (**A**) AK096174 expression was determined in SGC-7901 and BGC-823 cells transduced with empty vector, pCDNA-AK096174, sh-AK096174 1#, sh-AK096174 2#. (**B**,**C**) CCK-8 assays were used to determine the cell proliferation in SGC-7901 and BGC-823 cells, which were transfected with empty vector, pCDNA-AK096174, sh-AK096174 1#, sh-AK096174 2#. (**D**,**E**) The migratory and invasive abilities of the SGC-7901 and BGC-823 cells after transfecting with empty vector, pCDNA-AK096174, sh-AK096174 1#, sh-AK096174 2# were evaluated using Transwell assays. Scale bar = 50 μm. Data are presented as mean ± S.D. Experiments were independently conducted three times to obtain the presented data. *P<0.05 and **P<0.01.

The article "Long non-coding RNA AK096174 promotes cell proliferation and invasion in gastric cancer by regulating WDR66 expression" was retracted in 2023. Reasons: errors in the materials; errors in the data.

To determine the effect of AK096174 on cell proliferation, a CCK-8 assay was performed. As determined by CCK-8 assay, cell growth was inhibited when AK096174 expression was knocked down in SGC-7901 and BGC-823 cells compared with controls (Figure 2B,C). In contrast, overexpression of AK096174 could promote cell proliferation (Figure 2B).

To further determine whether AK096174 is associated with the progression of GC, we analyzed its effect on the migration and invasion of the BGC-823 and SGC-7901 cells. Using Transwell assay, we found that the BGC-823 and SGC-7901 cell migration and invasion were significantly impaired after the knockdown of AK096174 (Figure 2D,E). Conversely, AK096174 overexpression in these cells promoted cell migration and invasion (Figure 2D).

Furthermore, alteration of AK096174 led to differential expression of epithelial–mesenchymal transition (EMT) markers. Expression of the epithelial marker E-cadherin was increased, whereas expression of mesenchymal markers N-cadherin, Snail, and ZEB1 was decreased after AK096174 knockdown (Figure 3A–D). However, AK096174 overexpression in these cells up-regulated the expression of EMT markers (Figure 3A,B). Taken together, these findings indicate that AK096174 has important roles in GC progression.

**Figure 3:** The effect of AK096174 on cell EMT in gastric cell lines (**A**,**C**) Western blot analysis revealed the expression of E-cadherin, N-cadherin, Snail, and ZEB1 in SGC-7901 and BGC-823 cells, which were transfected with empty vector, pCDNA-AK096174, sh-AK096174 1#, sh-AK096174 2#. (**B**,**D**) Densitometry analysis depicts relative changes in the expression of E-cadherin, N-cadherin, Snail, and ZEB1. Data are presented as mean ± S.D. Experiments were independently conducted three times to obtain the presented data. *P<0.05 and **P<0.01.

### AK096174 functions as oncogene by up-regulating WDR66 expression in GC cells

It is widely accepted that lncRNA can regulate its neighboring protein-coding genes. AK096174 is located on the reverse strand of chromosome 12 (12q24.31). The *WDR66* gene is located less than 150 kb downstream of AK096174. Furthermore, some studies have shown that WDR66 is related to cancer and cancer metastasis. Thus, we hypothesized that WDR66 may be regulated by AK096174. To test this hypothesis, we performed real-time RT-PCR and Western blot to detect the transcription and protein level of WDR66 upon AK096174 knockdown or overexpression. Forty-eight hours after transfection, we examined the mRNA level of WDR66 in cells and we did not find significant variation in SGC-7901 and BGC-823 cells (Figure 4A). However, the protein level of WDR66 was significantly decreased by AK096174 knockdown and increased by AK096174 overexpression, suggesting that WDR66 is up-regulated by AK096174 at the translational level (Figure 4B). To provide further evidence that AK096174 promotes GC cells proliferation, migration, and invasion through regulating WDR66 expression, we knocked down the expression of WDR66 by siRNAs (Figure 4C). As expected, we found that introduction of si-WDR66 1# remarkably attenuated the cell proliferation, migration, invasion, and EMT induced by AK096174 overexpression (Figure 4D–F).

The article "Long non-coding RNA AK096174 promotes cell proliferation and invasion in gastric cancer by regulating WDR66 expression" was retracted in 2023. Reasons: errors in the materials; errors in the data.

**Figure 4:** AK096174 functions as oncogene by up-regulating WDR66 expression in gastric cell lines (**A**,**B**) The mRNA and protein levels of WDR66 were detected by real-time PCR and Western blot in SGC-7901 and BGC-823 cells, which were transfected with sh-AK096174, pCDNA-AK096174, or empty vector. (**C**) The mRNA level of WDR66 was detected by real-time PCR in SGC-7901 and BGC-823 cells, which were transfected with si-WDR66 or si-NC. (**D**) CCK-8 assays were used to determine the cell proliferation in SGC-7901 and BGC-823 cells, which were transfected with empty vector, pCDNA-AK096174, or co-transfected with pCDNA-AK096174 and si-WDR66. (**E**) Transwell assays were used to evaluate the migratory and invasive abilities of the SGC-7901 and BGC-823 cells after transfection with empty vector, pCDNA-AK096174, or co-transfected with pCDNA-AK096174 and si-WDR66. (**F**) Relative changes in the protein expression of E-cadherin, N-cadherin, Snail, and ZEB1 in the SGC-7901 and BGC-823 cells after transfection with empty vector, pCDNA-AK096174, or co-transfected with pCDNA-AK096174 and si-WDR66 were evaluated using Western blot. Scale bar = 50 μm. Data are presented as mean ± S.D. Experiments were independently conducted three times to obtain the presented data. *P<0.05 and **P<0.01.

In addition, to further confirm whether WDR66 is involved in GC cells proliferation, migration, and invasion, rescue assays were performed. We forcefully expressed WDR66 in SGC-7901 and BGC-823 cells by transfecting with WDR66 expression vector using the pCDNA vector (Figure 5A). The results revealed that co-transfection of pCDNA-WDR66 and sh-AK096174 1# could reverse the effects of down-regulated AK096174 on GC cells proliferation, migration, and invasion (Figure 5B,C), as well as EMT processes (Figure 6A,B). All these data indicated that AK096174 function as oncogene through targetting WDR66.

**Figure 5:** Forced expression of WDR66 promotes cell proliferation, migration, and invasion in gastric cell lines (**A**) The protein level of WDR66 were detected by real-time PCR and Western blot in SGC-7901 and BGC-823 cells, which were transfected with empty vector, sh-AK096174 1# or co-transfected with sh-AK096174 1# and pCDNA-WDR66. (**B**) CCK-8 assays were used to determine the cell proliferation in SGC-7901 and BGC-823 cells, which were transfected with empty vector, sh-AK096174 1#, or co-transfected with sh-AK096174 1# and pCDNA-WDR66. (**C**) Transwell assays were used to evaluate the migratory and invasive abilities of the SGC-7901 and BGC-823 cells after transfection with empty vector, sh-AK096174 1#, or co-transfected with sh-AK096174 1# and pCDNA-WDR66. Data are presented as mean ± S.D. Experiments were independently conducted three times to obtain the presented data. *P<0.05 and **P<0.01.

The article "Long non-coding RNA AK096174 promotes cell proliferation and invasion in gastric cancer by regulating WDR66 expression" was retracted in 2023. Reasons: errors in the materials; errors in the data.

**Figure 6:** Forced expression of WDR66 promotes cell EMT in gastric cell lines (**A**) Western blot analysis revealed the expression of E-cadherin, N-cadherin, Snail, and ZEB1 in SGC-7901 and BGC-823 cells, which were transfected with empty vector, sh-AK096174 1#, or co-transfected with sh-AK096174 1# and pCDNA-WDR66. (**B**) Densitometry analysis depicts relative changes in the expression of E-cadherin, N-cadherin, Snail, and ZEB1. Data are presented as mean ± S.D. Experiments were independently conducted three times to obtain the presented data. *P<0.05, **P<0.01, #*P*<0.05 and ##*P*<0.01.

## Discussion

Recently, RNA sequencing has revealed that hundreds of lncRNAs are dysregulated in several human cancers, indicating that lncRNAs are critical regulators during tumorigenesis and cancer progression [14–16]. In this study, we identified a novel oncogenic lncRNA: AK096174. We demonstrated that AK096174 expression was up-regulated in GC tissues and cell lines. Moreover, higher AK096174 expression was associated with a shorter OS of GC patients, indicating the pathological importance of AK096174 in tumor progression. Subsequently, we explored the biological function of AK096174 in GC by a series of molecular and cellular experiments *in vitro*. We found that knockdown of AK096174 in GC cells significantly inhibited cell proliferation, migration and invasion, and suppressed EMT through regulation of E-cadherin, N-cadherin, ZEB1, and Snail. In contrast, overexpression of AK096174 had promoting effects. Finally, we investigated the underlying mechanism of AK096174 in GC cells. We found that AK096174 could regulate WDR66 expression in GC cells. These results indicate that AK096174 may play an oncogenic role in the development of GC.

Invasion and metastasis are the main causes of cancer-related mortality, and EMT is well known to increase the motility and invasiveness of cancer cells [17,18]. Many recent studies have demonstrated that lncRNAs are involved in these processes and could influence the invasiveness of GC cells. For example, HOTAIR and H19 are classic oncogenic lncRNAs have proved that could promote cell invasion in multiple types of GC cells [19,20]. In addition, lncRNA-SNHG20, a newly identified GC, was found to regulate MKN45 and BGC-823 cells proliferation, invasion, and EMT by binding to EZH2 and regulated the GSK-3β/β-catenin signaling pathway [21]. Similarly, in our study, EMT associated with invasion and migration of GC cells was clearly enhanced in an AK096174-dependent manner. We observed that AK096174 significantly induced cell migration and invasion capacities. As demonstrated by our Transwell assay experiment, there was a dramatic reduction in the number of migrating and invasion cells after si-AK096174 transfection, relative to controls, which suggests that knockdown of AK096174 may inhibit invasiveness of GC cells. Furthermore, expression of EMT-promoting proteins, such as N-cadherin, Snail, and ZEB1, was significantly increased in AK096174-overexpressing cells. These results indicated that AK096174 could increase GC invasion and metastasis by promoting EMT.

The article "Long non-coding RNA AK096174 promotes cell proliferation and invasion in gastric cancer by regulating WDR66 expression" was retracted in 2023. Reasons: errors in the materials; errors in the data.

In our study, patients with high-AK096174 expression showed larger tumors, more frequent lymph node metastasis and advanced stage cancer. These conditions will eventually cause poor patient prognosis. However, high level of AK096174 failed to show association with DFS. We think that number of patients were too few to show significant difference in the present study. As survival rate is a more valuable parameter than lymphovascular invasion and lymph node involvement in clinical setting, further study including more patients is needed to solve this limitation.

When we explored the mechanisms by which AK096174 contributes to gastric carcinogenesis, we found the involvement of WDR66. The regulation of lncRNA on the expression of genes in close genomic proximity is called *cis*-acting regulation, which is a common regulatory mechanism of lncRNAs [22,23]. Thus, we searched the neighboring protein-coding genes near AK096174 on chromosome 12 to find potential target genes which AK096174 might influence. We found that the *WDR66* gene was located on the same strand within 150 kb downstream of AK096174. WD-repeat protein family is a large family found in all eukaryotes and is implicated in a variety of functions ranging from signal transduction and transcription regulation to cell cycle control, autophagy, and apoptosis [24]. A recent study found that high WDR66 expression was significantly associated with poor OS of patients suffering from esophageal squamous carcinomas (ESCC) [25]. Moreover, knockdown of WDR66 suppresses cell growth and motility and decreases EMT of ESCC cells [25]. Consistent with this study, we show that AK096174 can regulate WDR66 at translational level and that WDR66 is functionally responsible for AK096174-mediated gastric carcinogenesis. The specific biological mechanism by which AK096174 regulates WDR66 still needs to be further investigated.

The article "Long non-coding RNA AK096174 promotes cell proliferation and invasion in gastric cancer by regulating WDR66 expression" was retracted in 2023. Reasons: errors in the materials; errors in the data.

In conclusion, we demonstrated that AK096174 was up-regulated in GC tissues and cell lines. In addition, we demonstrated for the first time that down-regulation of AK096174 restricted cell proliferation and metastasis *in vitro*. We also showed that AK096174 could regulate WDR66 expression in GC cells. Our findings indicated AK096174 as a likely therapeutic target in the treatment of GC. However, whether the high expression of AK096174 is specific to GC or also to other types of cancer is still unclear and further study is needed to clarify this.

## Supporting information

## Abbreviations

CCK-8: cell counting kit 8
DFS: disease-free survival
EMT: epithelial–mesenchymal transition
ESCC: esophageal squamous carcinoma
GC: gastric cancer
lncRNA: long non-coding RNA
OS: overall survival
WDR66: WD repeat-containing protein 66
